# The Protective Effects of miR-21-Mediated Fibroblast Growth Factor 1 in Rats with Coronary Heart Disease

This article has been retracted.

**DOI:** 10.1155/2021/3621259

**Published:** 2021-12-01

**Authors:** Bin Zhang, Hongguang Liu, Guoping Yang, Yongmei Wang, Yan Wang

**Affiliations:** ^1^Department of Cardiology, Affiliated Hospital of Taishan Medical College, China; ^2^Department of Cardiology, Liaocheng Third People's Hospital, China; ^3^Department of Cardiology, Zhoucun District People's Hospital of Zibo City, China; ^4^Department of Cardiology, Tai'an Central Hospital, China; ^5^Department of Cardiology, Qingdao Central Hospital, China

## Abstract

**Aim:**

The study is to verify the protective effects of miR-21-mediated fibroblast growth factor 1 (FGF1) against myocardial ischemia in rats with coronary heart disease.

**Materials and Methods:**

Sprague-Dawley (SD) rat models of myocardial ischemia/reperfusion (MI/R) injury were constructed, and the expression of miR-21 and FGF1 in them was interfered through ischemic postconditioning. The protective effects of miR-21-mediated FGF1 on myocardium of the model rats were analyzed, and the targeted regulatory relationship between miR-21 and FGF1 was verified through myocardial cell experiments to find the mechanism of miR-21.

**Results:**

MiR-21 and FGF1 with increased expression could protect the cardiac function of model rats and improve their diastolic blood pressure (DBP), systolic blood pressure (SBP), heart rate (HR), coronary flow (CF), bax, and bcl-2 levels, but it would also cause further increase of vascular endothelial growth factor (VEGF) and decreased infarct size (INF). In addition, intervention through both miR-21 mimics and recombinant human FGF1 could highlight the above changes. Pearson correlation analysis revealed that the expression of miR-21 was positively correlated with that of FGF1, and both miR-21 and FGF1 were significantly and linearly correlated with DBP, SBP, HR, CF, INF, bax, and bcl-2, but they were not significantly correlated with the VEGF level. The myocardial cell experiment results revealed that upregulation of miR-21 or FGF1 could alleviate apoptosis caused by hypoxia/reoxygenation of myocardial cells, and inhibition of the FGF1 expression could hinder the effect of miR-21 against apoptosis of myocardial cells. Dual luciferase reporter assay revealed that transfection of miR-21-mimics could effectively raise the fluorescence intensity of pmirGLO-FGF1-3′UTR Wt but had no significant effect on that of pmirGLO-FGF1-3′UTR Mut.

**Conclusion:**

MiR-21 can specifically mediate the expression of FGF1 to relieve MI/R injury, protect the cardiac function, and resist apoptosis.

## 1. Introduction

Cardiovascular diseases are the major causes of death and disability worldwide, contributing to 30% of the global mortality and 10% of global burden of disease (1, 2). With the global population increase and population aging, from 1990 to 2013, the number of patients dead for cardiovascular diseases increased by 41% (3), of which about 8,200,000 people died of ischemic heart disease every year (4). Interruption of cardiac blood supply will seriously damage myocardial cells. Although interventional therapy can greatly help to restore cardiac coronary perfusion, but contradictorily, the reperfusion will further damage myocardium, and interventional therapy is unable to rebuild microvascular circulation (5, 6).

MicroRNAs (miRNAs), a kind of short-chain noncoding RNA with 20 bp-long nucleotides, widely exist in animals and plants, which regulates mRNA translation by binding to the 3′ untranslated region targeting mRNA, so it plays an important role in cardiovascular diseases including heart failure (7, 8). miRNAs also play an important role in development of myocardial cells and their survival under stress conditions (9). Previous research results revealed that miR-21 was involved in myocardial ischemia/reperfusion (MI/R) injury, and the protection mechanism of trimetazidine against MI/R injury was its promotion to the expression of miR-21 (10). In addition, the verification results of animal models also revealed that miR-21 could protect the cardiac function of rats with cardiac ischemia injury and reduce myocardial cell apoptosis of them (11). It can also protect the endothelial cells through phosphatase gene/vascular endothelial growth factor (VEGF) pathway (12). Fibroblast growth factor 1 (FGF1) is an important regulator of angiogenesis, which directly acts on myocardial cells to maintain the integrity of myocardial function and structure (12). Recently, it was reported that there were targeted binding sites between miR-21 and FGF1, and miR-21 could promote chondrocyte proliferation and suppress apoptosis of them by inhibiting the expression of FGF1 (13).

Whether the interaction between miR-21 and FGF1 in chondrocytes also exists in cardiomyocytes and whether the interaction affects the protective effects of miR-21 and FGF1 against myocardial ischemia injury and reperfusion are still under investigation. In order to find it, this study carried out the following analysis.

## 2. Materials and Methods

### 2.1. Establishment of Rat Models of Ischemia-Reperfusion (I/R)

A total of 60 mature Sprague-Dawley (SD) rats (strain code: 101; SCXK (Hu): 2017-0011) were all adaptively fed with general nutritious feedstuff (Beijing Zhecheng Technology Co., Ltd.) for one week after being purchased from Beijing Vital River Laboratory Animal Technology Co., Ltd., and the rats were fasted overnight and allowed to drink freely. Among the 60 rats, 40 of them were selected by the random number table method to prepare rat models of MI/R (14), and 10 of them were selected as a control group (CON group) and not intervened through surgery. The rest 10 rats were taken as a Sham operation group (Sham group) and intervened with thoracotomy to separate vessels but no operations about ischemia and perfusion. The 40 rats were intraperitoneally injected with pentobarbital sodium (Sigma, St. Louis, USA, 40 mg/kg) and ventilated with a positive pressure ventilator (ALC-V8, Shanghai, China). Before surgery, the tail clip test was used to check the sufficiency of anesthesia. Thorax was opened at the fourth intercostal space to free the left anterior descending coronary artery (LAD), and ligation was performed at the junction of left auricle and the site 1-2 mm below the boundary of pulmonary cone. The LAD was clamped for 30 minutes and then released for 120 minutes. The 40 model rats were divided into a model group (model group), a miR-21 mimics treatment group (miR-21 group), a FGF1 treatment group (FGF1 group), and a miR-21 mimics+ FGF1 treatment group (combination group) using the random number table method. During the release period of LAD, rats in the miR-21 group were treated with 100 *μ*L of 50 mg/kg miR-21 mimics through intramuscular injection at 10 different sites in the anterior wall of the left heart after being pretreated with liposome 2000, and rats in the FGF1 group were given recombinant human FGF1 through intravenous drip at 10 *μ*g/kg for 10 minutes. The miR-21 mimics was designed and synthesized by Shanghai Gene Pharma Co., Ltd., and recombinant human FGF1 (item number: 13241013) was purchased from the Thermo Fisher Scientific.

### 2.2. Electrophysiological Measurement of Rats

An electrophysiological signal recorder (Avante Trading (Beijing) Co., Ltd.) was employed to determine the diastolic blood pressure (DBP), systolic blood pressure (SBP), heart rate (HR), and coronary flow (CF) at the left ventricular of each rat in each group.

### 2.3. Measurement of Infarct Size

The living rats were executed by cervical dislocation after being measured fully, and their myocardial infarct size (INF) was measured based on cardiac tissues sampled from the rats using the computer planimetric method by referring to the method provided by Sodha et al. (15)

### 2.4. Construction and Transfection of Expression Vectors

All expression vectors were designed and synthesized by Shanghai Gene Pharma Co., Ltd., including miR-21 mimics, si-FGF1, sh-FGF1, pmirGLO-FGF1-3′UTR wild type (Wt), pmirGLO-FGF1-3′UTR mutant type (Mut), and blank vector, pmirGLO-NC. At 24 h before transfection, the cells were digested with trypsin, and then, the cells were transfected with expression vectors when the cell fusion reached about 80% according to specific operation steps in the kit instructions. Subsequently, the cells were cultured in an incubator with 5% CO_2_ at 37°C for 48 h, and the culture medium was replaced every 6 h. Quantitative real time polymerase chain reaction (qRT-PCR) was adopted to determine the transfection results. Cells not transfected were used as a control group. The Lipofectamine TM2000 transfection kit (item number: 35050) was purchased from the Invitrogen Company in the United States.

### 2.5. Grouping and Processing

Myocardial cells were separated from the heart of newborn SD rats (age ≤ 3 days) and cultured by referring to the method proposed by Sadoshima et al. (16), and they were determined using the specific labeling immunofluorescence staining. The cells were divided into a normal cell group, a cell model group, a miR-21 mimic group, a sh-FGF1 group, and a miR-21 mimics+ si-FGF1 group. Myocardial cells in the later three groups were transfected with miR-21 mimics, sh-FGF1, and miR-21 mimics+ si-FGF1, respectively.

### 2.6. Myocardial Cell Model

Myocardial cells were subject to hypoxic treatment under 3%O_2_, 5%CO_2_, and 92%N_2_ for 24 hours and then were reoxygenated under 5%CO_2_ and 95% air for 3 hours.

### 2.7. qRT-PCR

The total RNA was extracted from myocardial tissues and myocardial cells using TRIzol reagent, respectively, and the purity, concentration, and integrity of the total RNA were determined using a ultraviolet spectrophotometry and through agarose gel electrophoresis. The A260/A280 value between 1.8 and 2.1 was considered to meet the experimental requirements. The first strand cDNA was synthesized according to the kit instructions, and then, polymerase chain reaction (PCR) amplification was performed through a PCR system that consisted of 20 *μ*L of the total volume containing 0.4 *μ*L of upstream and downstream primers, respectively, 10 *μ*L of 2 × TransTaq® Tip Green qPCR SuperMix, 0.4 *μ*L of Passive Reference Dye (50x), and ddH2O to adjust the volume under predenaturation at 95°C for 30 s followed by 40 cycles of denaturation at 95°C for 5 s, and annealing and extension at 60°C for 30 s. The primer sequences are shown in Table 1.

### 2.8. Dual Luciferase Reporter Assay

Myocardial cells were transfected with pmirGLO-FGF1-3′UTR Wt, pmirGLO-FGF1-3′UTR Mut, miR-21-mimics, and miR-NC, respectively, after they were cultured to logarithmic growth phase. At 48 h after transfection, the fluorescence intensity of them was detected using the dual luciferase determination system.

### 2.9. Cell Apoptosis Determination

The cells were digested with 0.25% trypsin. After digestion, the cells were washed with PBS two times and then added with 100 *μ*L of binding buffer to prepare 1∗10^6^ cells/mL suspension. The suspension was added with AnnexinV-FITC and PI in order, incubated at room temperature for 5 min in the dark, and finally detected using the CytoFLE S flow cytometer system. The experiment was repeated three times, and the average value was taken. Annexin V-FITC/PI apoptosis determination kit (item number: V35113) was purchased from the Invitrogen Company in the United States.

### 2.10. Statistical Analysis

SPSS19.0 (Asia Analytics Formerly SPSS, China) was adopted for statistical analysis. Comparison between two groups was carried out using the *t*-test, while comparison among multiple groups was performed using the Analysis of Variance. Post hoc analysis was carried out by the LSD test, and correlation analysis was conducted using the Pearson correlation analysis. *P* < 0.05 indicated a significant difference.

## 3. Results

### 3.1. Protective Effects of miR-21 and FGF1 against MI/R Injury

As shown in Figure 1, the CON group was not different from the Sham group in the levels of DBP, SBP, HR, CF, VEGF, bax, and bcl-2 (all *P* > 0.05), and both groups showed no myocardial infarction. However, compared with the CON group and the Sham group, the model group showed increased DBP and HR (both *P* < 0.05), decreased SBP and CF (both *P* < 0.05), and large area of myocardial infarction, and it also showed increased VEGF and bax levels and decreased bcl-2 level in myocardial tissues (all *P* < 0.05). Rats intervened with miR-21 mimics, or recombinant human FGF1 showed improved levels of DBP, SBP, HR, bax, and bcl-2 (all *P* < 0.05) and also showed further improvement of VEGF and decrease in INF (both *P* < 0.05). Meantime, the intervention of both miR-21 mimics and recombinant human FGF1 contributed to more significant changes (*P* < 0.05).

### 3.2. The Expression of miR-21 and FGF1 in Myocardial Tissues

We determined the expression of miR-21 and FGF1 in myocardial tissues of rats in each group to find out whether the intervention was successful. It was turned out that the CON group was not different from the Sham group in the expression of miR-21 and FGF1 (both *P* > 0.05), but compared with the CON group and the Sham group, the model group showed decreased expression of them (*P* < 0.05). In addition, after being intervened with miR-21 mimics, SD rats in the model group showed increased expression of miR-21 and FGF1 in their myocardial tissues (both *P* < 0.05), but after being intervened by recombinant human FGF1, they only showed increased expression of FGF1 (*P* < 0.05), and after being intervened by the two factors meantime, they were not very different from those in the miR-21 group in the expression of miR-21 (*P* > 0.05) but showed significant higher expression of FGF1 than those in the FGF1 group (*P* < 0.05) (Figure 2)

### 3.3. Correlation Analysis

Pearson correlation analysis revealed that the expression of miR-21 was positively correlated with that of FGF1 (*P* < 0.05), and miR-21 and FGF1 were significantly and linearly correlated with DBP, SBP, HR, CF, INF, bax, and bcl-2 (all *P* < 0.05) but were not significantly correlated with the VEGF level (*P* > 0.05) (Figure 3)

### 3.4. The Role of miR-21 in Reducing Myocardial Cell Apoptosis by Targeting FGF1

The myocardial cell experiment results revealed that upregulation of miR-21 or FGF1 could alleviate apoptosis of myocardial cells caused hypoxia/reoxygenation (*P* < 0.05), and inhibition of the FGF1 expression could hinder the effect of miR-21 against apoptosis of myocardial cells (*P* < 0.05) (Figure 4)

### 3.5. Dual Luciferase Reporter Assay

The results of fluorescence intensity determination revealed that transfection of miR-21-mimics could effectively raise the fluorescence intensity of pmirGLO-FGF1-3′UTR Wt (*P* < 0.05) but had no significant effect on that of pmirGLO-FGF1-3′UTR Mut (*P* > 0.05) (Figure 5)

## 4. Discussion

Myocardial infarction is one of the five major manifestations of coronary heart disease. Thrombolytic therapy and interventional therapy are currently the main methods to alleviate myocardial ischemia injury in clinical practice. However, myocardial reperfusion will cause more serious injury or death, and MI/R injury is also an important influencing factor for poor prognosis of patients with coronary heart disease (17, 18). With the development of therapeutic drugs and methods, myocardial reperfusion has been continuously improved, but there is still a lack of effective means to prevent MI/R injury (19). The results of this study revealed that miR-21 could mediate FGF1 to protect myocardium of rats under ischemia reperfusion and reduce myocardial cell apoptosis, which may become a therapeutic target for preventing MI/R injury in the future.

We constructed rat models of MI/R injury by clamping and then releasing LAD. As we expected, all electrophysiological indexes of the heart of each rat were abnormal, including decreased SBP and CF and increased DBP and HR. Based on dissection of the rats, a large area of myocardial infarction was found, and it was also found that the myocardial tissues of the rats showed significantly lowered expression of miR-21 and FGF1, increased VEGF and bax levels, and lowered expression of bcl-2. It indicated that myocardial cell apoptosis was enhanced, but the rats also underwent ischemic preconditioning, and the VEGF expression promoted angiogenesis and maintained cardiac blood supply. During the recovery of blood supply in rats, we interfered the expression of miR-21 and FGF1 in the rats. The increase in the expression of miR-21 and FGF1 in myocardial cells of the rats suggested that we had successfully intervened it. Meantime, compared with the model rats not intervened, the rats showed some significantly improved cardiac function indexes, decreased myocardial INF, lowered level of the apoptosis factor, bax, and increased levels of antiapoptosis factors, bcl-2, and VEGF. It indicated that both miR-21 and FGF1 could intensity the resistance of myocardium against apoptosis caused by MI/R injury to protect cardiac function, and the simultaneous intervention of miR-21 and FGF1 could bring a more significant result. Correlation analysis results also revealed that miR-21 and FGF1 were significantly and linearly correlated with cardiac function, INF, bax, and bcl-2 in rats. Although our results showed that both miR-21 and FGF1 could promote the VEGF expression, we did not find any correlation between them. We speculated that it may be related to the self-resistance of rats against I/R injury. In this pathological process, many factors contribute to the increase of VEGF expression level to adapt to myocardial infarction. In addition, we also found that the expression of miR-21 had a significant positive correlation with that of FGF1. In order to verify whether there is an expression regulation relationship between miR-21 and FGF1, we extracted myocardial cells from neonatal rats and cultured them. It was turned out that downregulation of FGF1 expression could inhibit miR-21 from protecting myocardial cells from the injury caused by hypoxia/reoxygenation. Dual luciferase reporter assay revealed that miR-21 could targetedly promote the expression of FGF1 in myocardial cells. Therefore, based on these results, it can be concluded that miR-21 can targetedly mediate the expression of FGF1 to alleviate MI/R injury, protect cardiac function, and resist apoptosis.

Many previous studies reported that miR-21 could protect myocardial tissues from ischemia and reperfusion, and many downstream targets of miR-21 have been found, such as programmed cell death factor 4 (PDCD4). MiR-21/PDCD4 pathway can protect myocardial cells and weaken apoptosis caused by oxidative stress injury (20). In addition, miR-21 can regulate the TLR4/NF-*κ*B pathway to reduce the release of inflammatory factors and relieve myocardial cell injury during MI/R injury in rats (21). In addition to I/R injury in myocardium, miR-21 is also closely related to that in the kidney and brain (22, 23). Generally, miR-21 decreases during I/R injury, but the increase of it can protect organs by mainly reducing apoptosis and inhibiting the release of inflammatory factors. Vascular regeneration and microcirculation reconstruction are very important for the treatment of myocardial infarction. Many studies also reported that miR-21 was related to vascular regeneration, and overexpression of miR-21 could activate hypoxia-inducible factor 1*α* to promote neovascularization during limb ischemia reperfusion injury (24). FGF1 is also bound up with angiogenesis. Garbayo et al. (25) pointed out that intramyocardial injection of FGF1 could improve the cardiac function of pig models of ischemia reperfusion and promote angiogenesis.

However, miR-21 and FGF1 may play different roles in different cells. As mentioned earlier, Liu et al. (13) concluded that miR-21 suppressed the apoptosis of growth plate chondrocytes and promoted proliferation by targetedly inhibiting FGF1. Moreover, miR-21 may not entirely beneficial against MI/R injury. A study concluded that miR-21 targeted Smad 7 to promote myocardial fibrosis after myocardial infarction, and Smad 7 could regulate tumor necrosis factor beta signal transduction (26, 27). FGF1 is a profibrogenic factor. For example, it promotes pulmonary fibrosis and liver fibrosis (28, 29). However, there is no report on the relationship between FGF1 and myocardial fibrosis, which needs further research and analysis. In addition, the intervention method adopted in this study is ischemic postconditioning, and the role of ischemic preconditioning intervention has not been verified. We will further improve our analysis in future studies. As this is a single/limited region study, a multiregional or multicentric approach may provide a broad picture which can further enhance the validity of the prospective results. So far, not many efforts have been directed towards establishing a significant association between some of the circulatory candidate miRNAs and the severity of CAD when developing a noninvasive diagnostic method that can help in reducing coronary complications. Considering CAD as a multifactorial and multigenic disease driven by various genetic and nongenetic factors, observations from the current study appear to support the assumption that miRNA signatures have important implications on CAD and its different stages.

To sum up, miR-21 can targetedly mediate the expression of FGF1 to relieve MI/R injury, protect cardiac function, and resist apoptosis.

## Figures and Tables

**Figure 1:** Protective effects of miR-21 and FGF1 against MI/R injury: (a) changes of DBP in rats; (b) changes of SBP in rats; (c) changes in HR in rats; (d) changes of CF in rats; (e) changes of INF in rats; (f) changes of VEGF in rats; (g) changes of bax in rats; (h) changes of bcl-2 in rats. A: in comparison with the CON group, *P* < 0.05; B: in comparison with the Sham group, *P* < 0.05; C: in comparison with the model group, *P* < 0.05; D: in comparison with the miR-21 group, *P* < 0.05; E: in comparison with the FGF1 group, *P* < 0.05. DBP: diastolic blood pressure; SBP: systolic blood pressure; HR: heart rate; CF: coronary flow.

**Figure 2:** The expression of miR-21 and FGF1 in myocardial tissues: (a) changes of miR-21 in rats; (b) changes of FGF1 in rats. A: in comparison with the CON group, *P* < 0.05; B: in comparison with the Sham group, *P* < 0.05; C: in comparison with the model group, *P* < 0.05; D: in comparison with the miR-21 group, *P* < 0.05; E: in comparison with FGF1, *P* < 0.05. CON: control group.

**Figure 3:** Correlation analysis: (a) analysis of correlation between miR-21 and FGF1; (b) analysis of correlation between miR-21 and DBP; (c) analysis of correlation between miR-21 and SBP; (d) analysis of correlation between miR-21 and HR; (e) analysis of correlation between miR-21 and CF; (f) analysis of correlation between miR-21 and INF; (g) analysis of correlation between miR-21 and VEGF; (h) analysis of correlation between miR-21 and bax; (i) analysis of correlation between miR-21 and bcl-2; (j) analysis of correlation between FGF1 and DBP; (k) analysis of correlation between FGF1 and SBP; (l) analysis of correlation between FGF1 and HR. (m) analysis of correlation between FGF1 and CF; (n) analysis of correlation between FGF1 and INF; (o) analysis of correlation between FGF1 and VEGF; (p) analysis of correlation between FGF1 and bax; (q) analysis of correlation between FGF1 and bcl-2. DBP: diastolic blood pressure; SBP: systolic blood pressure; HR: heart rate; CF: coronary flow.

**Figure 4:** MiR-21 reduces myocardial cell apoptosis by targeting FGF1: (a) changes of miR-21 expression; (b) changes of FGF1 expression; (c) effects of miR-21 and FGF1 on myocardial cell apoptosis. A: in comparison with the normal group, *P* < 0.05; B: in comparison with the cell model group, *P* < 0.05; C: in comparison with the miR-NC group, *P* < 0.05; D: in comparison with the miR-21 minics group, *P* < 0.05; E: in comparison with the sh-FGF1 group, *P* < 0.05.

**Figure 5:** Dual luciferase reporter assay: (a) the expression of miR-21; (b) fluorescence intensity. A: in comparison with the CON group, *P* < 0.05; B: in comparison with the miR-NC group, *P* < 0.05. CON: control group.

**Table 1:** Primer sequences.

	Forward primer	Reverse primer
MiR-21	5′-GCGGCAACACCAGTCGATG-3′	5′-TGCGTGTCGTGGAGTC-3′
U6	5′-GCGCGTCGTGAAGCGTTC-3′	5′-GTGCAGGGTCCGAGGT-3′

## Data Availability

The authors confirm that the data supporting the findings of this study are available within the article.
